The article "Retinal Degeneration in a Murine Model of Retinal Ischemia by Unilateral Common Carotid Artery Occlusion" was published in 2021. Journal: Biomed Res Int.

# Retinal Degeneration in a Murine Model of Retinal Ischemia by Unilateral Common Carotid Artery Occlusion

**DOI:** 10.1155/2021/7727648

**Published:** 2021-12-31

**Authors:** Deokho Lee, Ayaka Nakai, Yukihiro Miwa, Yohei Tomita, Naho Serizawa, Yusaku Katada, Yusuke Hatanaka, Kazuo Tsubota, Kazuno Negishi, Toshihide Kurihara

**Affiliations:** ^1^Laboratory of Photobiology, Keio University School of Medicine, Tokyo 160-8582, Japan; ^2^Department of Ophthalmology, Keio University School of Medicine, Tokyo 160-8582, Japan; ^3^Department of Ophthalmology, Nihon University School of Medicine, Tokyo 173-0032, Japan; ^4^Animal Eye Care, Tokyo Animal Eye Clinic, Tokyo 158-0093, Japan; ^5^Department of Ophthalmology, Harvard Medical School, Boston Children's Hospital, Boston, MA 02115, USA; ^6^Tsubota Laboratory, Inc., Tokyo 160-0016, Japan

## Abstract

Retinal degeneration is a progressive retinal damage in ocular vascular diseases. There are several reasons for this, such as occlusion of arteries or veins, diabetic retinopathy, or hereditary retinal diseases. To study pathological mechanisms of retinal degeneration, it is required to develop experimentally reproducible and clinically relevant models. In our previous studies, we developed a murine model of retinal hypoperfusion by unilateral common carotid artery occlusion (UCCAO) which mimics the pathophysiology of ocular ischemic syndrome (OIS) in humans, and described broad pathological mechanisms in the retina after UCCAO. However, there still remain missing pieces of the ocular pathologic process by UCCAO. In this study, we examined those unfound mechanisms. UCCAO was performed on adult mice. Ocular dysfunctions, histological deficits, and inflammation were examined after UCCAO, compared with sham-operated mice. Evaluation values were analyzed by electrophysiological, histological, and molecular biological methods. Eyelid drooping was permanently seen after UCCAO. Induction time point of acute reversible cataract under anesthesia was shortened. Retinal/visual dysfunctions were detected 2-4 weeks after UCCAO. Specifically, scotopic b-wave was more affected than a-wave, with the dysfunction of photopic b-wave. Impaired oscillatory potentials and visual evoked potential were constantly observed. Pathological Müller gliosis/inflammation was featured with NeuN-positive cell loss in the ganglion cell layer. Axial length, intraocular pressure, pupillary light reflex, and retinal pigment epithelium/choroidal thickness were not changed by UCCAO. A murine model of retinal ischemia by UCCAO can be useful for studying a series of degenerative process in the ischemic retina.

## 1. Introduction

Retinal degeneration is a leading cause of incurable vision loss. Retinal degeneration occurs in various ways including occlusion of arteries or veins, diabetic retinopathy, or hereditary retinal diseases [1–5]. Ocular ischemia, occurring when the blood/oxygen supply in the eye is inadequate, commonly leads to retinal degeneration [6]. Anatomically, ocular ischemia can be caused by occlusion of the ophthalmic artery, which is a branch of the internal carotid artery from the common carotid artery (CCA) [7]. In humans, ocular ischemic syndrome (OIS) is classified as one of the vision-threatening diseases caused by occlusion of the carotid artery [6]. There is no promising treatment for OIS, and even the pathological mechanism for retinal degeneration in OIS needs fundamental investigations.

The article "Retinal Degeneration in a Murine Model of Retinal Ischemia by Unilateral Common Carotid Artery Occlusion" was published in 2021. Journal: Biomed Res Int.

To date, there are limited experimental animal models for retinal degeneration in OIS. Using bilateral occlusions of CCAs, rats have been widely used for understanding the pathological mechanism for retinal degeneration in OIS [8–10]. Relatively, mice have not been commonly utilized, as there exist the limitations for the model development using bilateral occlusions of CCAs [11, 12]. Bilateral stenosis of CCAs was attempted in mice using tricky microcoils under limited conditions such as probably excluding dead mice during/after the surgery [13].

For those reasons, we previously developed a mouse model of OIS by unilateral common carotid artery occlusion (UCCAO) with a simple suturing technique and demonstrated several retinal degenerative features in a mouse model of OIS with the 100% survival rate [11, 14–16]. However, there still remain missing pieces of the pathologic process in the UCCAO-operated eye, such as axial length, intraocular pressure (IOP), pupillary light reflex (PLR), acute reversible cataract under anesthesia, ocular (retinal and visual) function, the retinal pigment epithelium (RPE)/choroidal condition, pathological Müller gliosis, and inflammation.

In this study, we examined those unfound mechanisms of retinal degenerative characteristics in UCCAO-operated adult mice and more comprehensively introduced a mouse model of retinal ischemia by UCCAO which can mimic the pathophysiology of OIS.

## 2. Materials and Methods

### 2.1. Animals

Adult (5-6 weeks old) male C57BL6 mice were obtained from CLEA Japan (Tokyo, Japan), housed (5-6 mice per cage) on a 12/12 h light-dark cycle, and fed ad libitum. All animal experiments were approved by Keio University School of Medicine IACUC (Institutional Animal Care and Use Committees, Ethics ID number: 16017) and adhered to the ARVO (Association for Research in Vision and Ophthalmology) statement and the ARRIVE (Animal Research: Reporting of In Vivo Experiments) guidelines.

The article "Retinal Degeneration in a Murine Model of Retinal Ischemia by Unilateral Common Carotid Artery Occlusion" was published in 2021. Journal: Biomed Res Int.

### 2.2. UCCAO

After randomization followed by acclimatization for a week, mice were subjected to UCCAO, as previously indicated [11, 14–16]. Briefly, anesthetized mice by a mixture of midazolam (40 *μ*g/100 *μ*L; Sandoz, Tokyo, Japan), medetomidine (7.5 *μ*g/100 *μ*L; Orion, Espoo, Finland), and butorphanol tartrate (50 *μ*g/100 *μ*L; Meiji Seika Pharma, Tokyo, Japan) (termed, MMB) were carefully lied on an operating table, and a neck incision was made to find the right CCA. The right CCA was firmly occluded twice with 6-0 silk sutures (Figure 1(a)) and cut between the two occluded sites. After this procedure, the incision was closed with sutures, and mice were allowed to recover in their cages under a heating pad for a day. For a sham surgery, mice received the same procedure except for the occlusion. To confirm the successful occlusion, eyelid drooping was examined by the naked eyes (Figure 1(b)). The number of mice per experiment, data points of the analyses, and inclusion and exclusion criteria for further analyses were determined based on our previous papers [11, 14–16].

### 2.3. Electroretinography (ERG) and Visual Evoked Potential (VEP)

Scotopic and photopic ERG was performed as previously indicated [14–16]. Mice were dark adapted more than 12 hours. After pupil dilation by a mixture of 0.5% tropicamide and phenylephrine as well as anesthesia by a mixture of MMB, mice were placed in a Ganzfeld dome with LED stimulators on the PuREC acquisition system (PuREC, MAYO, Inazawa, Japan). Active electrodes were placed to the contact lens. The amplitudes of ERG waveforms were measured at various flash intensities. VEP was performed as previously indicated [17]. Before 5 days of VEP, a mixture of MMB was injected to mice for anesthesia. Then, 2 stainless steel pan-head screws (M1.0 × 6.0 mm) were inserted to the mouse skull above the primary visual cortex (1.5 mm anterior and 1.5 mm lateral to lambda). On the day of VEP, anesthetized mice by a mixture of MMB were placed in a Ganzfeld dome with LED stimulators on the PuREC acquisition system (PuREC, MAYO, Inazawa, Japan). Active electrodes were placed on the screws. The amplitudes of ERG waveforms were measured at a 1 Hz 3 cd.s/m^2^ flash intensity.

### 2.4. Spectral Domain-Optical Coherence Tomography (SD-OCT)

Axial length and RPE/choroidal thickness were measured by SD-OCT (Envisu R4310, Leica, Wetzlar, Germany), as previously indicated [18]. After pupil dilation by a mixture of 0.5% tropicamide and phenylephrine as well as anesthesia by a mixture of MMB, mice were placed on an OCT platform to fix the mouse posture for SD-OCT scanning. Axial length was measured from the anterior corneal surface to the RPE line along the corneal vertex reflection line. As the choroidal thickness varies depending on the location of the eye, the choroidal area at 0.5 mm distant from the optic disc was calculated to compare the mean choroidal thickness between UCCAO-operated and sham-operated mice. The area of the circumference of RPE/choroid was quantified with the NIH ImageJ program (National Institutes of Health, Bethesda, MD, USA) [19]. Then, the area was divided by the circumference to determine the RPE/choroidal thickness.

The article "Retinal Degeneration in a Murine Model of Retinal Ischemia by Unilateral Common Carotid Artery Occlusion" was published in 2021. Journal: Biomed Res Int.

### 2.5. IOP, Acute Reversible Cataract, and PLR Measurements

IOP was measured, as previously indicated [17]. After pupil dilation by a mixture of 0.5% tropicamide and phenylephrine as well as anesthesia by a mixture of MMB, we placed a tonometer (TonoLab, Vantaa, Finland) near the contact lens and measured IOP. For the detection of acute reversible cataract, mice were firstly anesthetized by a mixture of MMB. Under anesthesia with or without pupil dilation by a mixture of 0.5% tropicamide and phenylephrine, the induction time point of cataract was checked every 5 minutes after 5 minutes of the injection of a mixture of MMB. For the PLR evaluation, freely behaving mice were fixed by hands and adjusted to provide the opportunity to acquire close-up images of the pupils in the acquisition system (Capture-Ex(GV) Version 3.10, Library Inc., Tokyo, Japan). Mice were dark adapted for 2 minutes. Images were recorded using an infrared CCD camera (BS-GV200, Library Inc., Tokyo, Japan) under the absence/presence of white LED light with the GW Instek power supply system. Based on the pupil images, PLR was grossly examined.

### 2.6. Immunohistochemistry (IHC)

IHC was performed as previously described [14–17]. For the preparation of retinal flat mounting samples, the eyeballs were enucleated and fixed with 4% paraformaldehyde (PFA). Then, the retinas from the eyeballs were obtained, simply flat mounted, and incubated with cold methanol. Then, the flat mounted retinas were rinsed with PBS several times, permeabilized with PBS containing 0.1% Triton X-100 and 0.1% BSA, and probed with isolectin GS-IB4 from *Griffonia simplicifolia* (IB4) conjugated with Alexa Fluor 488 (Invitrogen, Carlsbad, CA, USA) at 4°C overnight. After washing with PBS several times, the flat mounted retinas were mounted on microscope slides with cover glasses and examined via a fluorescence microscope (LSM710, Carl Zeiss, Jena, Germany). For the preparation of sagittal sectioning samples, the 4% PFA-fixed eyeballs were incubated in 30% sucrose until the eyeballs went to the bottom of the tube. Then, the eyeballs were embedded in O.C.T. compound (Sakura Tissue-Tek, Tokyo, Japan). Sagittal sectioning samples (12 *μ*m) were obtained using a cryostat (Leica CM3050S, Leica, Wetzlar, Germany). They were rinsed with PBS several times, permeabilized with PBS containing 0.1% Triton X-100 and 0.1% BSA, and probed with the following primary antibodies: anti-glial fibrillary acidic protein (GFAP) antibody (1 : 400, Cat #13–0300, Thermo Fisher Scientific, USA), anti-glutamine synthetase (GS) antibody (1 : 400, MAB302, Sigma-Aldrich, USA), and anti-NeuN antibody (1 : 400, Cat #ABN78; Sigma-Aldrich, USA). After washing with PBS several times, they were incubated with appropriate Alexa Fluor-conjugated secondary antibodies (Thermo Fisher Scientific, USA), and nuclei were stained with DAPI. Then, they were mounted with cover glasses and examined via a fluorescence microscope (LSM710, Carl Zeiss, Jena, Germany). The GFAP immunolabeling was quantified by a morphology score as previously described [11, 14, 16] (0: no signal, 1: labeled processes in the ganglion cell layer, 2: labeled processes in the inner retinal layer, and 3: labeled processes in the entire retinal layer). The number of immunolabeled cells was counted with the same method as previously described [14, 17].

The article "Retinal Degeneration in a Murine Model of Retinal Ischemia by Unilateral Common Carotid Artery Occlusion" was published in 2021. Journal: Biomed Res Int.

### 2.7. Western Blotting and Quantitative PCR

For western blotting, protein extraction, electrophoresis, and band visualization were performed as same as described in our previous literature [15, 16]. Antibodies used in this study are as follows: anti-HIF-1*α* (1 : 1000, Cat #36169, Cell Signaling Technology, Danvers, MA, USA) and anti-*β*-actin (1 : 5000, #3700, Cell Signaling Technology, MA, USA). For quantitative PCR, total RNA was extracted using a commercial kit (the RNeasy Plus Mini Kit, Qiagen, Venlo, The Netherlands), and its concentration was quantified using a spectrophotometer (NanoDrop 2000c, Thermo Scientific, Waltham, MA, USA). Then, total RNA was converted to cDNA using a commercial Kit (the ReverTra Ace qPCR RT Master Mix with gDNA Remover, TOYOBO, Osaka, Japan). Quantitative PCR was performed with a SYBR green master mix commercial kit (THUNDERBIRD SYBR® qPCR Mix, TOYOBO, Osaka, Japan) using a PCR system (the Step One Plus Real-Time PCR system, Applied Biosystems, Waltham, MA, USA). Primer sequences for the current study are listed in Table 1. The fold difference in different transcripts was calculated by the *ΔΔ*CT protocol.

### 2.8. Fluorescein Isothiocyanate- (FITC-) Dextran Labeling and Laser Speckle Flowmetry (LSF)

FITC-dextran labeling was performed as previously indicated [20, 21] with minor modifications. After anesthesia by a mixture of MMB, 150 *μ*L of FITC-dextran (12.5 mg/ml, 2000 kD, Sigma, USA) was injected into the left ventricles of mice. After systemic circulation for 1.5 minutes, mice were sacrificed, and the eyeballs were enucleated. The flat mounted retinas were obtained from the eyeballs, incubated with cold methanol, mounted on microscope slides with cover glasses, and photographed with a fluorescence microscope (BZ-9000, KEYENCE, Osaka, Japan). Images of the whole retina were collected at 10x magnification and merged into one image using the BZ-II Analyzer system (KEYENCE, Osaka, Japan). For measuring relative cerebral blood flow (CBF), LSF (Omegazone OZ-2 mini, Omegawave, Inc., Tokyo, Japan) was used as previously indicated [22–24] with minor modifications. Recordings were performed under anesthesia with MMB. The skull was exposed by a midline incision of the scalp. Then, illumination of infrared laser was conducted to the skull surface, followed by detection of the scattered light using a CCD camera over the head. Signal processing with detected signals was performed with the LSF imager (Omegazone OZ-2 mini, Omegawave, Inc., Tokyo, Japan), and the calculated values were considered CBF [25].

The article "Retinal Degeneration in a Murine Model of Retinal Ischemia by Unilateral Common Carotid Artery Occlusion" was published in 2021. Journal: Biomed Res Int.

### 2.9. Statistical Analysis

All experimental values were presented as mean ± standard deviation. The data were analyzed by blinded investigators as much as possible, using the computer-based software package Prism 5 (GraphPad, San Diego, CA, USA). *P* value < 0.05 was considered statistically significant.

## 3. Results

### 3.1. General Screening of Pathophysiological Ocular Changes by UCCAO

As the induction of ocular ischemia in the right eye by the occlusion of the right CCA was expected (Figure 1(a)), the right eye of UCCAO-operated mice and sham-operated mice was used and further analyzed in this current study. Right after UCCAO, we found the droopy eyelid in all the mice (Figure 1(b)). Eyelid drooping was permanent during the whole experimental period. For the general screening of pathophysiological ocular alterations by UCCAO, currently available parameters such as axial length, acute reversible cataract, PLR, and IOP were investigated (Figures 1(c)–1(f)). There was no significant change in axial length between UCCAO-operated and sham-operated mice (Figure 1(c)). When it comes to acute reversible cataract under anesthesia, we found that the induction time point of cataract was significantly shortened in UCCAO-operated mice under any conditions with-and-without pupil dilation (Figure 1(d)). Significant differences in PLR and IOP were not observed between UCCAO-operated and sham-operated mice (Figures 1(e) and 1(f)).

Next, as UCCAO has been described to have abnormalities in retinal blood circulation analyzed by FITC-dextran angiography [11, 21], we also examined blood perfusion in the retina with the same method (Figure 2(a)). Right after UCCAO, a complete perfusion of FITC-dextran was observed in the sham-operated retina, while FITC-dextran labeling was not filled yet in the UCCAO-operated retina. As induction of hypoxia/ischemia could be examined by a general hypoxic marker (HIF-1*α*) [26], HIF-1*α* expression was examined in the retina a day after UCCAO (Figure 2(b)). As expected, HIF-1*α* expression significantly increased in the UCCAO-operated retina. On the other hand, we attempted to examine whether the central nervous system (especially, the brain) could also be affected (Figure 2(c)). A slight reduction in relative CBF was significantly detected in the right middle cerebral artery core region right after UCCAO. Hypoxia-responsive gene expressions were further screened in the retina on day 1 after UCCAO (Figure 2(d)). We found that *Vegf* and *Bnip3* mRNA expressions significantly increased in the UCCAO-operated retina even though fold changes were not dramatic. The mRNA expressions of the other genes (*Epo*, *Glut1*, and *Pdk1*) showed increasing tendencies without statistical significance. When it comes to RPE/choroid in UCCAO-operated mice, *Bnip3* mRNA expression significantly increased with small extent. *Epo* mRNA expression showed increasing tendencies without statistical significance, while any changes in *Glut1* and *Pdk1* expressions were not observed.

The article "Retinal Degeneration in a Murine Model of Retinal Ischemia by Unilateral Common Carotid Artery Occlusion" was published in 2021. Journal: Biomed Res Int.

### 3.2. Ocular Dysfunction and Ganglion Cell Loss after UCCAO

Retinal functional changes were examined after UCCAO (Figures 3 and 4). The amplitudes of OPs significantly decreased in UCCAO-operated mice, compared to those in sham-operated mice on week 2 after UCCAO (Figures 3(a) and 3(b)). While the amplitude of scotopic a-wave was not significantly changed (Figure 3(c)), the amplitude of scotopic b-wave significantly decreased in UCCAO-operated mice on week 2 after UCCAO (Figure 3(d)). The amplitude of photopic b-wave also significantly decreased in UCCAO-operated mice on week 2 after UCCAO (Figures 3(e) and 3(f)). We could see the permanent damage on retinal function after UCCAO (Figure 4). Decreases in the amplitudes of OPs, scotopic b-wave, and photopic b-wave were constantly seen on week 4 after UCCAO (Figures 4(a), 4(b), and 4(d)–4(f)), while the amplitude of scotopic a-wave was not dramatically changed (Figures 4(a) and 4(c)). As scotopic b-wave was continuously more damaged than scotopic a-wave, the relative ratio of b/a-wave was calculated using the values on weeks 2 and 4 after UCCAO (Figure 4(g)). The reduction in the relative ratio of b/a-wave was detected after UCCAO.

Next, visual functional changes were examined after UCCAO (Figures 5(a) and 5(b)). The amplitude of VEP significantly decreased on week 2 and week 4 after UCCAO. As b-wave was more affected than a-wave in UCCAO-operated mice (Figures 3 and 4), we further examined whether inner retinal degeneration occurs after UCCAO (Figure 5(c)). We found that the number of NeuN-positive cells in the ganglion cell layer significantly decreased on week 2 after UCCAO (Figure 5(c)). As a-wave was not dramatically affected in UCCAO-operated mice (Figures 3 and 4), we examined whether the RPE/choroidal thickness was changed by UCCAO (Figure 5(d)). There was no significant difference in the RPE/choroidal thickness between UCCAO-operated and sham-operated mice 2 and 4 weeks after UCCAO (Figure 5(d)).

The article "Retinal Degeneration in a Murine Model of Retinal Ischemia by Unilateral Common Carotid Artery Occlusion" was published in 2021. Journal: Biomed Res Int.

### 3.3. Retinal Müller Gliosis and Inflammation after UCCAO

Pathological Müller gliosis occurs in retinal ischemic processes [27, 28]. Previously, pathological gliosis has been described acutely and chronically after UCCAO [11, 14, 16]. Based on the morphology of cells only stained by GFAP in the ischemic retina, Müller gliosis was presumably considered. Therefore, we examined whether Müller gliosis could be seen after UCCAO (Figure 6(a)). GFAP-stained morphology scoring in the UCCAO-operated retina was significantly higher than that in the sham-operated retina, and double labeling of GFAP/GS (one of the representative Müller cell markers [29, 30]) was clearly observed (Figure 6(a)).

Next, as IB4 staining has been simply used for the labeling of inflammatory cells [31, 32], we used this strategy to screen inflammatory processes in the ischemic retina after UCCAO (Figure 6(b)). We found that the number of IB4-positive inflammatory cells significantly increased in the UCCAO-operated retina (Figure 6(b)). Furthermore, we screened the induction of several inflammatory cytokines/chemokines in the ischemic retina after UCCAO (Figure 6(c)). *Ccl2* mRNA expression showed increasing tendencies after UCCAO with wide extent, while changes in the mRNA expressions of *Ccl12* and *Cox-2* were not dramatic without any statistical significance (Figure 6(c)).

## 4. Discussion

Our current study was designed to understand whether UCCAO could induce a series of retinal degenerative processes in the ischemic retina, which has not yet been found in previous studies using a murine model of retinal ischemia by UCCAO [11, 14–16]. Furthermore, we reported what could not be observed in UCCAO-operated adult mice by screening of several pathophysiological parameters such as axial length, IOP, and PLR, which have not also been tested yet. In this study, we enabled more comprehensive understanding of an experimental model of retinal ischemia by UCCAO in adult mice. This is significance of our current study.

The article "Retinal Degeneration in a Murine Model of Retinal Ischemia by Unilateral Common Carotid Artery Occlusion" was published in 2021. Journal: Biomed Res Int.

The carotid artery is the most important blood vessel in humans as it is the line between the life and death. As the carotid artery helps transport most of blood into the central nervous system (the brain as well as the eye) [33], ocular ischemia could occur by stenosis or occlusion of the carotid artery [3]. Anatomically, the eye is supplied by the ophthalmic artery, which is the first branch of internal carotid artery from the CCA [7]. Therefore, theoretically, stenosis of occlusion of the CCA could clearly induce ocular ischemia. However, well-developed collateral circulation has chances to prevent this phenomenon in humans [6, 34]. Experimentally, to induce ocular ischemia, bilateral occlusions of CCAs were applied to adult rats due to their well-developed collateral circulation [8–10]. Adult black mice (C57BL/6) could not be subjected to bilateral occlusions of CCAs in that they die during/after the surgery [11, 20], of which outcome is related to a lack of the complete Circle of Willis in adult black mice (especially, the missing of the posterior communicating artery) [35–37]. In other words, however, unilateral occlusion of CCA could be enough to induce ocular ischemia in adult black mice. Then, how about the other strains of mice? It would be interesting to perform a comparison study on ocular ischemic stresses by UCCAO in different strains of mice, as similar as a comparison study conducted in 1997 on cerebral ischemic stresses by BCCAO in several mouse strains [12].

In our study, retinal damages were more detected than choroidal damages in UCCAO-operated mice. Retinal photoreceptors (rods and cones) are mainly suggested as the origin of a-wave, while bipolar cells and/or Müller cells have been considered as the origin of b-wave [38–43]. OPs are largely generated from various inner retinal cells including bipolar cells, amacrine cells, and ganglion cells [44–46]. VEP provides information about the entire visual pathway, from the retina to the visual cortex [47, 48]. In this regard, decreases in the amplitudes of b-wave, OPs, and VEP without a dramatic change in the amplitude of a-wave may be partially explainable under the pathological condition of the UCCAO-operated eye. Nonetheless, from the anatomical point of view, RPE/choroid could also be affected as the choroidal plexus is derived from the ophthalmic artery [7]. In clinical cases, chronic choroidal thinning was detected in some individual patients with OIS [49–51]. For cardiovascular diseases including OIS, metabolic abnormalities are commonly accompanied to narrow walls of the carotid arteries [52, 53]. In fact, atherosclerosis is the major cause of OIS [3, 54]. This should be considered to understand the discrepancy between clinical cases for OIS and our UCCAO mouse model. Taken together, more investigations on RPE/choroidal damages by UCCAO or UCCAO with metabolic disorders in adult black mice need to be studied to clearly mimic the clinical condition of OIS.

The article "Retinal Degeneration in a Murine Model of Retinal Ischemia by Unilateral Common Carotid Artery Occlusion" was published in 2021. Journal: Biomed Res Int.

In UCCAO-operated mice, acute reversible cataract rapidly appeared under anesthesia. The inevitable development of anesthesia-induced acute reversible cataract has been described in experimental animals for a long time [55–57]. Even though the formation mechanism (plausibly explained with dried corneal surface, lowered body temperature, and hypertonic osmolarity [55–57]) as a side effect of anesthetic drugs in experimental animals have not been clearly understood, at least, it appears to be associated with marked alterations in the physiological state of the eye. In this regard, we assume that the UCCAO-operated eye may be more vulnerable to the anesthesia-induced disruption of physiological balance in the eye. We further demonstrated that all UCCAO-operated mice had permanent eyelid drooping in our current and previous studies as well as the others [11, 15, 58]. The droopy eyelid has been indicated as one of the representative signs of neurological disorders and diseases [59]. The levator palpebrae superioris (the muscle responsible for maintaining the eyelid position) is supplied by the lateral palpebral artery, a branch of the ophthalmic artery [60]. It also supports the notion that the disruption of physiological balance occurs in the ischemic eye by UCCAO.

Retinal ischemia, degeneration, inflammation, and pathological Müller gliosis were observed after UCCAO. As retinal ischemia is commonly accompanied with a series of these conditions (experimentally and clinically) [61–64], we think that a murine model of UCCAO also showed similar outcomes in the retina. Previously, we demonstrated that UCCAO induced HIF-1*α* stabilization in the eye [11, 15]. Along with reproducing that result in this study, we further found hypoxia-responsive gene induction (especially, *Bnip3* and *Vegf* in the retina and *Bnip3* in the RPE/choroid) after UCCAO. BNIP3 is one of the mitochondrial proteins related to activation of cell death pathways [65]. Previously, we demonstrated HIF-1*α*/BNIP3 pathway could be associated with inner retinal degeneration in a murine model of retinal ischemia/reperfusion injury by a transient induction of high IOP [17]. Inner retinal cell loss analyzed with NeuN staining was featured in the UCCAO-operated eye in this study, and apoptosis analyzed with terminal deoxynucleotidyl transferase dUTP nick end labeling (TUNEL) staining was seen in the inner retina of the UCCAO-operated eye in our previous study [14]. In this regard, we assume that retinal cell death could be seen in the UCCAO-induced ischemic retina through HIF-1*α*/BNIP3 pathway. This notion will be further studied in this murine model of retinal ischemia by UCCAO. Moreover, increases in inflammatory cells and *Ccl2* mRNA expression as well as pathological Müller gliosis were observed in the UCCAO-induced ischemic retina at the same time. CCL2, also known as monocyte chemotactic protein 1, is one of the key chemokines that could regulate migration and infiltration of monocytes at the systemic level [66]. In the retina, induction of CCL2 has been widely featured in various eye diseases including age-related macular degeneration, diabetic retinopathy, and retinopathy of prematurity [67–71]. Taken together, a murine model of retinal ischemia by UCCAO could also be used for studying the fundamental role of CCL2 in the development and progression of ischemia-mediated retinal inflammation. Previously, we found that the more pathological retinal gliosis occurs, the more the impairment of OPs is observed [16]. Inner retinal degeneration could be associated with pathological Müller gliosis in the UCCAO-induced ischemic retina. In this regard, our murine model of retinal ischemia by UCCAO could be applicable to understand how pathological Müller gliosis affects retinal function in the ischemic retina, which has not been yet clearly studied.

The article "Retinal Degeneration in a Murine Model of Retinal Ischemia by Unilateral Common Carotid Artery Occlusion" was published in 2021. Journal: Biomed Res Int.

## 5. Conclusions

In this study, we introduced a mouse model of retinal ischemia by UCCAO which can mimic the pathophysiology of OIS with changes of various ischemic parameters. Even though more investigations on the relationships between the ischemic retina, optic nerve damage, and ischemic brain (especially, the visual cortex) are highly intriguing in UCCAO-operated mice as they are interconnected, we ensure at this point that a murine model of retinal ischemia by UCCAO is highly applicable to study the pathophysiology of OIS and screen promising drug candidates for ischemic retinopathies.

## Figures and Tables

**Figure 1:** General characteristics of a murine model of retinal ischemia induced by unilateral common carotid artery occlusion (UCCAO). (a) A schematic illustration of the surgical procedure for UCCAO. UCCAO was performed by permanent suturing of the right common carotid artery (CCA). ICA: internal carotid artery; ECA: external carotid artery. Gray box, the cutting area. (b) Representative images of permanent eyelid drooping after UCCAO. (c) There was no significant change in axial length on week 2 (W2) and week 4 (W4) after UCCAO (*n* = 5 per group). *P* > 0.05. (d) A representative image of acute reversible cataract under medetomidine, midazolam, and butorphanol- (MMB-) induced anesthesia. The induction time point of acute reversible cataract in UCCAO-operated mice was shorter than that in sham-operated mice under MMB-induced anesthesia with-and-without pupil dilation (*n* = 8‐12 per group). ^∗^*P* < 0.05 and ^∗∗^*P* < 0.01. (e) Representative images of pupillary light reflex (PLR). The gross observation indicated that PLR was normal in UCCAO-operated mice under the dark/light condition, similar with that in sham-operated mice (*n* = 5‐6 per group). (f) There was no significant change in intraocular pressure (IOP) on day 0 (D0, right after UCCAO), week 2 (W2), and week 4 (W4) after UCCAO (*n* = 5‐8 per group). *P* > 0.05. The data were analyzed using Student's *t*-test (two-tailed) and presented as mean ± standard deviation.

The article "Retinal Degeneration in a Murine Model of Retinal Ischemia by Unilateral Common Carotid Artery Occlusion" was published in 2021. Journal: Biomed Res Int.

**Figure 2:** Abnormal retinal perfusion after UCCAO. (a) Whole retinal and optic nerve head (ONH) images showed that there was less perfusion in the retina right after UCCAO, detected with circulation of 2000 kD fluorescein isothiocyanate- (FITC-) dextran (12.5 mg/ml, 150 *μ*L) through the left ventricle of mice for 1.5 minutes (*n* = 3 per group). Scale bar, 1000 and 500 (ONH) *μ*m. (b) HIF-1*α* stabilization was seen in the retina a day after UCCAO (*n* = 4 per group). (c) A decrease in relative cerebral blood flow (CBF) was seen in the skull over the right (R) middle cerebral artery core region (dotted circles) right after UCCAO (*n* = 4 per group), analyzed with LSF. Ant: anterior; Mid: midline. (d) There were significant increases in hypoxia-responsive genes in the UCCAO-operated retina and RPE/choroid in comparison with those in the sham-operated retina and RPE/choroid a day after UCCAO, respectively (*n* = 5 per group). ^∗^*P* < 0.05 and ^∗∗^*P* < 0.01. The data were analyzed using Student's *t*-test (two-tailed) and presented as mean ± standard deviation. CH: choroid.

**Figure 3:** Retinal dysfunction 2 weeks after UCCAO. (a) Representative waveforms of scotopic a-wave, b-wave, and oscillatory potentials (OP1-4) responsive to a stimulus intensity of 10 cd.s/m^2^ 2 weeks after UCCAO. (b) The amplitudes of scotopic OPs in the UCCAO-operated eyes significantly decreased compared to those in the sham-operated eyes (*n* = 5 per group). ^∗^*P* < 0.05 and ^∗∗^*P* < 0.01. (c, d) The amplitude of scotopic b-wave (not scotopic a-wave) in the UCCAO-operated eyes significantly decreased compared to that in the sham-operated eyes (0.5 and 10 cd.s/m^2^) (*n* = 5 per group). ^∗^*P* < 0.05. (e) Representative waveforms of photopic b-wave responsive to a stimulus intensity of 20 cd.s/m^2^ 2 weeks after UCCAO. (f) The amplitude of photopic b-wave in the UCCAO-operated eyes significantly decreased compared to that in the sham-operated eyes (4 and 20 cd.s/m^2^) (*n* = 5 per group). ^∗^*P* < 0.05. The data were analyzed using Student's *t*-test (two-tailed) and presented as mean ± standard deviation.

The article "Retinal Degeneration in a Murine Model of Retinal Ischemia by Unilateral Common Carotid Artery Occlusion" was published in 2021. Journal: Biomed Res Int.

**Figure 4:** Retinal dysfunction 4 weeks after UCCAO. (a) Representative waveforms of scotopic a-wave, b-wave, and oscillatory potentials (OP1-4) responsive to a stimulus intensity of 10 cd.s/m^2^ 4 weeks after UCCAO. (b) The amplitudes of scotopic OPs in the UCCAO-operated eyes significantly decreased compared to those in the sham-operated eyes (*n* = 7 per group). ^∗∗^*P* < 0.01 and ^∗∗∗^*P* < 0.001. (c, d) The amplitude of scotopic b-wave (not scotopic a-wave) in the UCCAO-operated eyes significantly decreased compared to that in the sham-operated eyes (0.5 and 10 cd.s/m^2^) (*n* = 7 per group). ^∗^*P* < 0.05. (e) Representative waveforms of photopic b-wave responsive to a stimulus intensity of 20 cd.s/m^2^ 4 weeks after UCCAO. (f) The amplitude of photopic b-wave in the UCCAO-operated eyes decreased compared to that in the sham-operated eyes (4 and 20 cd.s/m^2^) (*n* = 7 per group). ^∗^*P* < 0.05 and ^∗∗^*P* < 0.01. (g) The relative ratio of b/a-wave was calculated using the values in Figures 3(c) and 3(d) and (c, d) (10 cd.s/m^2^). ^∗∗^*P* < 0.01. The data were analyzed using Student's *t*-test (two-tailed) and presented as mean ± standard deviation.

**Figure 5:** Visual dysfunction and ganglion cell loss after UCCAO. (a, b) Representative waveforms of visual evoked potential (VEP) responsive to a stimulus intensity of 3 cd.s/m^2^. The amplitude of VEP in the UCCAO-operated eyes significantly decreased compared to that in the sham-operated eyes on week 2 (W2) and week 4 (W4) after UCCAO (3 cd.s/m^2^) (*n* = 5 per group). ^∗^*P* < 0.05. (c) Representative images and quantitative analyses showed that the number of NeuN-positive cells in GCL of UCCAO-operated mice significantly decreased compared with that in GCL of sham-operated mice 2 weeks after UCCAO (*n* = 5 per group). ^∗∗^*P* < 0.01. GCL: ganglion cell layer; INL: inner nuclear layer; ONL: outer nuclear layer. White dotted squares, enlarged images. Scale bar, 100 and 50 (enlarged) *μ*m. (d) Representative images and quantitative analyses showed there was no significant change in the RPE/choroidal thickness on week 2 (W2) and week 4 (W4) after UCCAO (*n* = 5 per group). *P* > 0.05. Scale bar, 200 *μ*m. The data were analyzed using Student's *t*-test (two-tailed) and presented as mean ± standard deviation.

**Figure 6:** Retinal Müller gliosis and inflammation after UCCAO. (a) Representative images and quantitative analyses showed that morphology scoring stained by GFAP with GS (referred to as Müller gliosis) in UCCAO-operated mice was significantly higher compared with that in sham-operated mice 2 weeks after UCCAO (*n* = 4‐5 per group). ^∗^*P* < 0.05. GCL: ganglion cell layer; INL: inner nuclear layer; ONL: outer nuclear layer. Asterisk, glial activation. White dotted squares, enlarged images. Scale bar, 100 and 40 (enlarged) *μ*m. (b) Representative images and quantitative analyses showed that the number of IB4-positive inflammatory cells in UCCAO-operated mice significantly increased compared with that in sham-operated mice 2 weeks after UCCAO (*n* = 6 per group). ^∗∗^*P* < 0.01. Asterisk, IB4-positive inflammatory cells. White dotted squares, enlarged images. Scale bar, 100 and 50 (enlarged) *μ*m. (c) There were increasing tendencies and a significant increase in *Ccl2* mRNA expression in the UCCAO-operated retina in comparison with that in the sham-operated retina for 4 weeks after UCCAO, respectively. ^∗^*P* < 0.05. There was no significant change in the other genes (*Ccl12* and *Cox-2*) on week 1 (W1), week 2 (W2), and week 4 (W4) after UCCAO (*n* = 5‐6 per group). *P* > 0.05. The data were analyzed using Student's *t*-test (two-tailed) and presented as mean ± standard deviation. IB4: isolectin GS-IB4 from *Griffonia simplicifolia*.

The article "Retinal Degeneration in a Murine Model of Retinal Ischemia by Unilateral Common Carotid Artery Occlusion" was published in 2021. Journal: Biomed Res Int.

**Table 1:** Primer list.

Name	Direction	Sequence (5′→3′)	Accession number
*Hprt*	Forward	TCAGTCAACGGGGGACATAAA	NM_013556.2
	Reverse	GGGGCTGTACTGCTTAACCAG	

*Cox-2*	Forward	CAGACAACATAAACTGCGCCTT	NM_011198.4
	Reverse	GATACACCTCTCCACCAATGACC	

*Vegf*	Forward	CCTGGTGGACATCTTCCAGGAGTACC	AY707864.1
	Reverse	GAAGCTCATCTCTCCTATGTGCTGGC	

*Bnip3*	Forward	GCTCCCAGACACCACAAGAT	NM_009760.4
	Reverse	TGAGAGTAGCTGTGCGCTTC	

*Pdk1*	Forward	GGCGGCTTTGTGATTTGTAT	NM_172665.5
	Reverse	ACCTGAATCGGGGGATAAAC	

*Glut1*	Forward	CAGTTCGGCTATAACACTGGTG	NM_011400.3
	Reverse	GCCCCCGACAGAGAAGATG	

*Epo*	Forward	GGCCATAGAAGTTTGGCAAG	NM_007942
	Reverse	CCTCTCCCGTGTACAGCTTC	

*Ccl2*	Forward	CCCAATGAGTAGGCTGGAGA	NM_011333.3
	Reverse	TCTGGACCCATTCCTTCTTG	

*Ccl12*	Forward	GCTACAGGAGAATCACAAGCAGC	NM_011331.3
	Reverse	ACGTCTTATCCAAGTGGTTTATGG	

## Data Availability

The data is available on request to the corresponding author.
